The article "Artificial Intelligence Assistive Technology in Hospital Professional Nursing Technology" was published in 2021. Journal: J Healthc Eng.

# Artificial Intelligence Assistive Technology in Hospital Professional Nursing Technology

**DOI:** 10.1155/2021/1721529

**Published:** 2021-11-27

**Authors:** Yanxue Cai, Moorhe Clinto, Zhangbo Xiao

**Affiliations:** ^1^Second Affiliated Hospital, Qiqihar Medical University, Qiqihar 161006, China; ^2^Cuyahoga Community College, Cleveland, Ohio 43085, USA

## Abstract

Global aging is becoming more and more serious, and the nursing problems of the elderly will become very serious in the future. The article designs a control system with ATmega128 as the main controller based on the function of the multifunctional nursing robot. The article uses a convolutional neural network structure to estimate the position of 3D human joints. The article maps the joint coordinates of the colour map to the depth map based on the two camera parameters. At the same time, 15 joint heat maps are constructed with the joint depth map coordinates as the centre, and the joint heat map and the depth map are bound to the second-level neural network. The prediction of the position of the user's armpit is further completed by image processing technology. We compare this method with other attitude prediction methods to verify the advantages of this research method. The research background of this article is carried out in the context of global aging in the 21st century.

## 1. Introduction

In recent years, the problems of walking and movement of the elderly, the disabled, and others have received more attention from scientific researchers in various countries. Many countries have carried out scientific research in this field. Most research studies on human pose recognition focus on estimating 2D human joint coordinates from colour maps. The deep learning method based on large datasets has shown excellent results in detecting joint human points in colour images [1]. However, these algorithms cannot directly provide the position of the human body in the global coordinate system for the transfer and transportation care robot.

To ensure the accuracy of human body posture recognition of the transfer and transportation nursing robot, this paper uses the colour map human joint detection model as the first-level neural network to calculate the colour map human joint pixel coordinates. The article maps the joint coordinates of the colour map to the depth map based on the two camera parameters. At the same time, 15 joint heat maps are constructed with the joint depth map coordinates as the centre, and the joint heat map and the depth map are bound to the second-level neural network. Finally, this paper obtains the global coordinates of 15 joints. Artificial intelligence is a technology developed to simulate, extend, and expand human intelligence.

The article "Artificial Intelligence Assistive Technology in Hospital Professional Nursing Technology" was published in 2021. Journal: J Healthc Eng.

## 2. Transfer and Transportation Nursing Robot

Figure 1 shows the transfer and transportation nursing robot “Baize” developed by the team. The human-like back-carrying robot uses sound source localization, visual recognition, and other means to realize the position localization and posture recognition of the person cared for. The functions of autonomous obstacle avoidance and autonomous navigation are realized through the perception of the surrounding environment [2]. Tactile sensors are installed on the robot arm, chest rest, and seat to sense the user's back hug status in real time. The real-time safety guarantee module in the core control system adjusts the robot's movements and can safely and comfortably complete the actions of lifting, carrying, transferring, and placing. These designs provide intelligent transport services for groups with lower limb inconvenience. These all illustrate the application of artificial intelligence assistive technology in hospital professional nursing technology.

To achieve the above functions, the team designed the transfer and transportation nursing robot (Figure 2). The transfer nursing robot first uses the microphone array and the sound processing module to recognize the user's voice and calculates the user's angle relative to the robot to turn to the user. The human body gesture recognition module and the path planning module move to the user in front of the user at a short distance. Finally, the robot drives to the destination and places the user according to the guidance of the path plan.

## 3. Level 1 Convolutional Neural Network

According to the needs of the transfer and transportation nursing robot, this article defines the human joints as 15 joint points (Figure 3). The human body 3D joint position prediction is divided into a two-level network [3]. In the first-level network, we use PAF (part affinity field) to predict the state of the human body in the colour map. After calculating each pixel's human joint likelihood value, we take the maximum coordinate as the joint coordinate.

### 3.1. 2D Joint Point Detection

The PAF method has the characteristics of high precision and high robustness. It can effectively detect the 2D posture of the human body from the RGB image. This method uses a 2D human joint detection model to generate a multichannel scoring heat map *S*_est_ ∈ *ℝ*^*n*×*m*×15^, *S*_est_=(*S*_0_, *S*_1_,…, *S*_*i*_,…, *S*_14_). We order *p*_*i*_=arg max_(*u*_*s*_, *v*_*s*_)_*S*_*i*_(*u*_*s*_, *v*_*s*_), where *u*_*s*_, *v*_*s*_ represents the coordinates of the heat map and *p*_*i*_ represents the coordinates of the maximum score value in the heat map *S*_*i*_, that is, the predicted pixel coordinates of the joint *i*. Then, we get the predicted coordinates *p*_est_=(*p*_0_, *p*_1_,…, *p*_*i*_,…, *p*_14_), *p*_est_ ∈ *ℝ*^2×15^, of 15 joints. To further improve the adaptability of the PAE method to the working environment of nursing robots, we use the weights provided by Open Pose as the initial weights. At the same time, we use the family environment dataset to perform migration learning on the network [4].

The article "Artificial Intelligence Assistive Technology in Hospital Professional Nursing Technology" was published in 2021. Journal: J Healthc Eng.

### 3.2. Loss Function

To predict the joint pixel positions, we define a 15-channel real heat map during model training. *S*_*gt*_ represents 15 Gaussian images with the real joint pixel position as the extreme centre. We calculate the minimum mean square error of *S*_*gt*_ and *S*_est_ as the loss function of model optimization:

(1) $$\begin{array}{c} L_{2D}=\frac{1}{15}\sum_{\left(u_{c},v_{c}.i\right)}\left\|S_{gt}\left(u_{c},v_{c},i\right)-S_{\text{est}}\left(u_{c},v_{c},i\right)\right\|. \end{array}$$

## 4. Joint Heat Map

This paper constructs a multichannel joint heat map with the pixel coordinates of the 15 human joint point depth maps as the centre. We first calculate the depth map mapping relationship of the colour map to obtain the joint depth coordinates. The article obtains the denoising depth map:

(2) $$\begin{array}{c} I_{\text{depth}}\left(u_{\text{depth}},v_{\text{depth}}\right)=\text{med}\left\{D\left(u_{\text{depth}}-k,v_{\text{depth}}-l\right)\right\},k,l\in W, \end{array}$$

where (*u*_depth_, *v*_depth_) represent the pixel coordinates of the depth map; *k*, *l* represent the values in the template *W*; and med stands for median operation. Considering that the pixel coordinates of the depth map can be mapped to the camera coordinate system, this paper maps the *I*_depth_ pixel to the colour map *I*_color_ to obtain the two-picture pixel coordinate registration relationship map *M*_reg_. In this way, the coordinates of the joint depth map can be calculated in reverse [5]. The process is as follows.

**Step 1 .**

The article obtains *I*_depth_, *I*_color_,  and *M*_reg_ at the same time. Add 2 channels based on the colour image *I*_color_. These channels are used to store the corresponding depth map pixel coordinates. Define the coordinate of the pixel *x*_depth_ in *I*_depth_ as (*u*_depth_, *v*_depth_).

**Step 2 .**

Construct a 3-dimensional vector *p*_depth_=(*u*_depth_, *v*_depth_, *z*) for pixel *x*_depth_, where *z* is the pixel value of *I*_depth_ at *x*_depth_.

**Step 3 .**

Calculate the coordinate *p*_depth_^∼^ of *x*_depth_ in the depth camera coordinate system through the depth camera internal parameter matrix *H*_depth_ and *p*_depth_.

(3) $$\begin{array}{c} p_{\text{depth}}^{∼}=H_{\text{depth}}^{-1}p_{\text{depth}}. \end{array}$$

**Step 4 .**

The article "Artificial Intelligence Assistive Technology in Hospital Professional Nursing Technology" was published in 2021. Journal: J Healthc Eng.

The article uses the space coordinate transformation matrix to transform *p*_depth_^∼^ into the coordinate *p*_color_^∼^ in the colour camera coordinate system.

(4) $$\begin{array}{c} p_{\text{color}}^{∼}=p_{\text{depth}}^{∼}+T, \end{array}$$

where *R*, *T* represent the rotation matrix and translation matrix between the two cameras, respectively.

**Step 5 .**

Calculate the corresponding coordinate *p*_color_ of *x*_depth_ in the colour image coordinate system through the colour camera internal parameter matrix *H*_color_ and the colour camera coordinate system coordinate *p*_color_^∼^.

(5) $$\begin{array}{c} p_{\text{color}}=H_{\text{color}}p_{\text{color}}^{∼}. \end{array}$$

Repeat the above calculation for each pixel in *I*_depth_ in turn to obtain the coordinates of the mapped colour map. In this way, the pixel coordinates of the depth map corresponding to the pixel coordinates of each colour map can be obtained in reverse. Finally, we get the *R* − *G* − *B* − *U*_depth_ − *V*_depth_ five-channel registration image *M*_reg_.

**Step 7 .**

Find the joint depth map coordinate *p*_est_depth_ corresponding to the joint colour map coordinate *p*_est_ according to *M*_reg_. We define the multichannel joint heat map *H*=(*H*_0_, *H*_1_,…, *H*_*i*_,…, *H*_14_),  with *i* as the joint index [6]. The *H*_*i*_ dimension of the heat map is the same as the *I*_depth_ dimension. *p*_*h*_=(*u*_*h*_, *v*_*h*_) is the pixel coordinate of the heat map. We use the 1-dimensional Gaussian function *h*()() to calculate *H*_*i*_ with the coordinate *p*_est_depth_ of the joint depth map as the centre:

(6) $$\begin{array}{c} H_{i}\left(u_{h},v_{h},i\right)=g\left(\left\|p_{h}-p_{\text{est\_depth}}\left(i\right)\right\|\right). \end{array}$$

## 5. Level 2 Convolutional Neural Network

In the second stage, we use depth image and multichannel joint heat map binding as input. We further optimize the 2D joint detection results through convolutional neural networks to obtain 3D human joint poses. The algorithm flow is shown in Figure 4.

### 5.1. Network Structure

The real-time human posture recognition algorithm based on a 3D convolutional network relies on a high-performance GPU (graphics processing unit), which is unsuitable for ordinary households' transfer and transportation care robot systems [7]. Therefore, to meet the accuracy requirements of joint prediction, especially near-range joint prediction, this paper uses a compromised 2D convolution method instead of 3D convolution. Based on the VGG16 network structure and the spatial pyramid pooling method (SPP), we design a convolutional neural network that is not limited by the size of the input image (Figure 5). We replace the 1000-unit fully connected layer final output by VGG16 with a 45-unit fully connected layer. The *u* − *v* − *z* coordinates of 15 joints are estimated to get *p*_est_depth_^∼^=(*p*_est_depth_^0^, *p*_est_depth_^1^,…, *p*_est_depth_^*i*^,…, *p*_est_depth_^14^), *p*_est_depth_^∼^ ∈ *ℝ*^3×15^.

The article "Artificial Intelligence Assistive Technology in Hospital Professional Nursing Technology" was published in 2021. Journal: J Healthc Eng.

Defining the global coordinates is the same as defining the depth camera coordinates. The depth map camera coordinates *p*_est_depth_^*i*^ are converted to the global coordinates *p*_est_*w*_^*i*^ by formula (7), *p*_est_*w*_^*i*^=(*x*_*w*_^*i*^, *y*_*w*_^*i*^, *z*_*w*_^*i*^) is obtained, and then *p*_est_*w*_=(*p*_est_*w*_^0^,…, *p*_est_*w*_^*i*^,…, *p*_est_*w*_^14^) is obtained.

(7) $$\begin{array}{c} \left\{\begin{array}{c} x_{w}=z_{w}\frac{\left(u-u_{\text{cam}}\right)}{f_{x}},\\ y_{w}=z_{w}\frac{z_{w}\left(v-v_{\text{cam}}\right)}{f_{y}},\\ z_{w}=z. \end{array}\right. \end{array}$$

Among them, *f*_*x*_, *f*_*y*_, *u*_cam_, *v*_cam_ represent the internal camera parameters and *x*_*w*_, *y*_*w*_, *z*_*w*_ represent the coordinate values of the global coordinate system.

In this paper, based on the ITOP (invariant-top view) dataset, the application scenario data training network of the transfer and handling nursing robot is added.

### 5.2. Loss Function

We use the minimum mean square error between the predicted joint global coordinates and the actual joint global coordinates as the loss function of the second-level neural network:

(8) $$\begin{array}{c} L_{3D}=\frac{1}{15}\sum_{i=0}^{i=14}\left\|p_{\text{est}\_w}^{i}-p_{gt\_w}^{i}\right\|, \end{array}$$

where *i* is the joint index, *p*_est_*w*_^*i*^ is the predicted joint position, and *p*_*gt*_*w*_^*i*^ is the actual joint position.

## 6. Estimation of Underarm Points

We put the robot's two arms under the user's armpit which is the key to successfully picking up the user. This paper delineates ROI (region of interest) for the depth image based on the given depth image joint coordinates [8]. Then, we perform threshold segmentation in the ROI to obtain the underarm area and determine the target point where the robot arm is placed.

### 6.1. Pretreatment

We use the left (right) shoulder joint, left (right) elbow joint, and the midpoint of the left and right hip joints as vertices and delineate two triangles' ROIs. To ensure that the armpit area obtained by image segmentation does not contain the human body, we map the grey pixel value in the human body area to 1/3 of the original range [9]. We calculate the maximum depth *j*_max_ and minimum depth *j*_min_ among the four joint positions of the left (right) shoulder joint, left (right) elbow joint, left hip joint, and right hip joint in each ROI in turn. According to the pixel value mapping function shown in formula (9), the ROI is converted to grayscale.

(9) $$\begin{array}{c} \left\{\begin{array}{cc} p_{\text{out}}=p_{\text{in}}\text{,} & p_{\text{in}}<j_{\min},\\ p_{\text{out}}=\frac{1}{3}p_{\text{in}}+\frac{2}{3}j_{\min}, & j_{\min}\leq p_{\text{in}}<j_{\max},\\ p_{\text{out}}=p_{\text{in}}-\frac{1}{3}j_{\max}+\frac{2}{3}j_{\min}, & j_{\max}\leq p_{\text{in}}. \end{array}\right. \end{array}$$

The article "Artificial Intelligence Assistive Technology in Hospital Professional Nursing Technology" was published in 2021. Journal: J Healthc Eng.

### 6.2. Estimation of Axillary Points

We first perform 5 × 5 median filter denoising processing on the depth map. Considering that the background and foreground depth values vary with the scene, this paper uses the Otsu segmentation algorithm based on the maximum between-class variance to obtain the mask image *M* of the armpit area [10]. Further, we calculate the pixel coordinate *p*_est_*sp*_ of the armpit centre point by the following formula:

(10) $$\begin{array}{c} p_{\text{est}\_sp}=\frac{\sum_{\left(i,j\right)}M\left(i,j\right)\times \left(i,j\right)}{\sum_{\left(i,j\right)}M\left(i,j\right)}. \end{array}$$

## 7. Experiments and Results

The PC configuration used in this experiment is Intel Core i7-6700HQ CPU, with 8G RAM and 4G NVIDIA GeForce GTX 950M GPU. The colour map and depth map sensors use the Microsoft Kinect 2 sensor. For the lower limb inconvenience group, we selected 1,100 human body images in the home environment as the test dataset.

### 7.1. Real-Time Evaluation

The experimental results of the calculation speed of commonly used gesture recognition methods are shown in Table 1. The comparison shows that the 3D convolution method used in [10] single-time 3D joint position estimation exceeds elapsed time 2 s. This cannot meet the real-time requirements of the transfer and handling nursing robot. Therefore, the follow-up experiments of this article will not be tested. The Kinect SDK v2.0 method can complete about 30 joint predictions per second. The real-time performance of the algorithm at this time is optimal. The method in [9] is similar to the method in a single calculation, and the time is about 200 ms. This can prove the good real-time performance of the method in this paper.

### 7.2. Average Accuracy Evaluation

We use the 10 cm rule as the evaluation criterion for joint prediction. The article adopts the average accuracy of joint prediction (mAP) to measure the accuracy of the method used. Under the condition that the distance between the user and the camera is 550 mm–3500 mm, we collect 600 pieces of actual work scene data of the transfer and transportation nursing robot. The results of our evaluation of Kinect SDK v2.0, the method of Fujisawa et al. [9], and this paper's method are shown in Figure 6.

The article "Artificial Intelligence Assistive Technology in Hospital Professional Nursing Technology" was published in 2021. Journal: J Healthc Eng.

It can be seen from Figure 6 that when we predict each joint of the human body, the average estimation accuracy of the KinectSDKv2.0 method is the lowest. The direct mapping method used in [9] has good environmental adaptability and high accuracy. However, due to the colour map, the joint estimation itself has certain errors. This method easily predicts failure in relatively slender parts such as hands, elbows, and knees. In addition, the method is also deeply affected by the invalid value of the depth map and the noise, which reduces the accuracy. Compared with the above methods, this method has the highest accuracy, and the average accuracy of joints reaches 91.5%.

### 7.3. Accuracy Evaluation at Close Range

We use the transfer and transportation care robot developed by our team. We collect 350 working environment datasets and evaluate the close-range robustness of the method in this paper under the short-distance conditions with the operating range of 550 mm–800 mm. This article only evaluates the estimation effect of each method on the near-distance joint estimation based on the coordinate prediction of the head, neck, left and right hips, left and right elbows, and left and right shoulders.

It can be seen from Figure 7 that all three methods have reached the highest estimation accuracy on the head. Kinect SDK v2.0 and [9] methods have the lowest estimation accuracy at the hip joint, while the method in this paper has the lowest estimation accuracy at the elbow joint. Overall, the estimation accuracy of this method in any joint is the highest among the three methods. The average accuracy of the joint reaches 90.3%. When the distance is between 550 mm and 800 mm, the human body information collected by the depth camera is not comprehensive. Compared with the average accuracy evaluation experiment, the accuracy of Kinect SDK v2.0 dropped sharply in the close-range experiment. The algorithm has misjudgement of joint positions and even misidentified joints that do not exist in the figure, which is unacceptable for the transfer and transportation nursing robot.

On the other hand, the depth camera based on the ToF (time of flight) principle is more sensitive to the wrinkles and colours of clothes under close-range conditions. In this way, it is easier to collect invalid values, which increases the probability of the direct mapping method [9] to map invalid values. This leads to an increase in the recognition error rate. In comparison, the two-stage network method proposed in this paper has better short-range adaptability.

The article "Artificial Intelligence Assistive Technology in Hospital Professional Nursing Technology" was published in 2021. Journal: J Healthc Eng.

### 7.4. Evaluation of the Accuracy of the Axillary Point Prediction

This article defines the 3 cm non-background rule as the basis for evaluating the accuracy of the axillary points. The predicted axillary point cannot be located on the human body, and the distance from the real axillary point in the *X-Y* plane is not more than 3 cm. It is regarded as an accurate prediction. Before calculating the user's armpit position, the transfer and transportation care robot moves to the front of the human body to face the front of the human body. We collect 150 frontal human body images at a distance of 550 mm–800 mm. Based on this, the experimental results of the evaluation of the method in this paper are shown in Figure 7.

After calculation, the method's accuracy for predicting the axillary points in this paper has reached 91.3%. This is because most of the operating objects are elderly people with mobility impairments under the conditions of transfer and transportation care applications. The human body is mostly in a passive state without too many complicated movements, and the body's posture is relatively simple. In addition, the method in this paper is based on human posture detection to obtain ROI. The prediction accuracy of the axillary points is directly related to the recognition ability of left (right) shoulder joint coordinates, left (right) elbow joint coordinates, and left (right) hip joint coordinates. Therefore, when the camera is too close to collect specific joint information, the armpit point estimation cannot be reliably completed when the joint position is incorrectly recognized.

## 8. Conclusion

This paper designs a 3D human pose estimation system for home care robots. The system uses Kinect 2 as the RGB-D data acquisition device to realize human joint position reasoning based on colour map 2D human body pose estimation. Through image processing technology, the prediction of the position of the user's axillary point is further completed. We compare this method with other posture prediction methods to verify the advantages of this research method and illustrate the correctness of the application of artificial intelligence assistive technology in hospital professional nursing technology [11, 12].

## Figures and Tables

**Figure 1:** The transfer and transportation care robot.

**Figure 2:** The control architecture of the transfer care robot.

**Figure 3:** Distribution of human joints.

**Figure 4:** Human pose recognition algorithm.

**Figure 5:** Level 2 neural network structure.

**Figure 6:** Comparison of average estimation accuracy.

**Figure 7:** Example of axillary point prediction.

**Table 1:** Operation time for gesture recognition.

	Kinect SDK v2.0	[9]	[10]	Method of this article
Single calculation time (ms)	33	180	2400	210

The article "Artificial Intelligence Assistive Technology in Hospital Professional Nursing Technology" was published in 2021. Journal: J Healthc Eng.

## Data Availability

The human body images data used to support the findings of this study are restricted by the Ethical Care Committee of Qiqihar Medical University in order to protect patient privacy. Data are available from Zhangbo Xiao (e-mail address: xzbmd@qmu.edu.cn) for researchers who meet the criteria for access to confidential data.
